# Kinematic Evaluation via Inertial Measurement Unit Associated with Upper Extremity Motor Function in Subacute Stroke: A Cross-Sectional Study

**DOI:** 10.1155/2021/4071645

**Published:** 2021-08-19

**Authors:** Ze-Jian Chen, Chang He, Ming-Hui Gu, Jiang Xu, Xiao-Lin Huang

**Affiliations:** ^1^Department of Rehabilitation Medicine, Tongji Hospital, Tongji Medical College, Huazhong University of Science and Technology, Wuhan, Hubei, China; ^2^World Health Organization Cooperative Training and Research Center in Rehabilitation, Wuhan, Hubei, China; ^3^Institute of Rehabilitation and Medical Robotics, State Key Lab of Digital Manufacturing Equipment and Technology, Huazhong University of Science and Technology, Wuhan, Hubei, China

## Abstract

Kinematic evaluation via portable sensor system has been increasingly applied in neurological sciences and clinical practice. However, conventional kinematic evaluation rarely extends the context beyond the motor impairment level. In addition, kinematic tasks with numerous items could be complex and time consuming that pose a burden to test applications and data processing. The study aimed to explore the correlation of finger-to-nose task (FNT) kinematics via Inertial Measurement Unit with upper limb motor function in subacute stroke. In this study, six FNT kinematic variables were used to measure movement time, smoothness, and velocity in 37 participants with subacute stroke. Upper limb motor function was evaluated with the Fugl-Meyer Assessment for Upper Extremity (FMA-UE), Action Research Arm Test (ARAT), and modified Barthel Index (MBI). As a result, mean velocity, peak velocity, and the number of movement units were associated with the clinical assessments. The multivariable linear regression models could estimate 55%, 51%, and 32% of variance in FMA-UE, ARAT, and MBI, respectively. In addition, age, gender, type of stroke, and paretic side had no significant effects on these associations. Results show that FNT kinematic variables measured via Inertial Measurement Unit are associated with upper extremity motor function in individuals with subacute stroke. The objective kinematic evaluation may be suitable for predicting clinical measures of motor impairment and capacity to understand upper extremity motor recovery and clinical decision making after stroke. This trial is registered with ChiCTR1900026656.

## 1. Introduction

Upper extremity (UE) motor function is impaired in approximately 50–80% of individuals with acute stroke [1] and 40–50% with chronic stroke [2, 3]. Motor impairment results in poor movement control and has a major impact on functional capacity and activities of daily living (ADL) of stroke survivors [4]. To optimize UE recovery after stroke, it is crucial to select multilevel outcome measures for the interpretation of motor recovery and clinical decision making [5]. Although there have been extensive validated UE scales or tests to assess body structure, function, and activity in clinical practice [6], these assessments often rely on subjectively rated ordinal scales with ceiling effects that may lead to examiner bias or lack sensitivity to detect potentially impactful changes of upper limb motor recovery [7].

Kinematic evaluation facilitates interpreting the mechanisms of motor restoration, which has been increasingly applied in neurological sciences and clinical practice [8–10]. Such technology is capable of providing detailed information regarding upper extremity function evaluation and delivering personalized interventions. According to the previous literature, kinematic assessment is usually performed using arm-supported robots or optical-camera systems, based on fixed laboratory environments or expensive equipment that leads to several disadvantages [11–13]. From the technical perspective, robotic instruments are unable to capture the entire spectrum of UE motor impairment due to their mechanical structure [14]. Moreover, most robotic devices could not extend the value of kinematic scenarios beyond the impairment level according to the International Classification of Functioning, Disability and Health (ICF) framework [11, 15]. Optical camera systems raise privacy concerns inevitably and constrain participants into a laboratory environment with much setup time and cost [16].

Portable sensor systems, a novel approach of kinematic evaluation, can provide upper limb spatiotemporal measurements against gravity in a natural three-dimensional environment [17]. Inertial Measurement Units (IMU) are portable sensor devices combining the three-dimensional accelerometers, gyroscopes, and magnetometers to detect kinematic parameters. Kinematic analysis of motor impairment via Inertial Measurement Unit has been shown to be objective, sensitive, and quantitative. However, kinematic tasks with numerous items could be complex and time consuming that pose burden on test application, compliance issues, and data processing in previous studies [18, 19]. Moreover, its relationship with the multilevel UE clinical measures regarding ICF framework has not been fully investigated [14, 20].

In clinical practice, the finger-to-nose test (FNT) is commonly applied to evaluate upper limb coordination in patients with stroke and cerebellar ataxia [12, 21]. Compared with multi-item clinical scales that require trained personnel and as long as 30 minutes to complete, FNT could reduce task burden when estimating individual's UE performance [22]. Previous studies have shown that FNT could add value to measure UE coordination with construct, convergent, and discriminant validity [12, 23] as well as ADL-related dexterity [24, 25]. However, it remains unclear how FNT correlates with motor impairment, capacity, and ADL performance in individuals with subacute stroke from a kinematic perspective. Therefore, the purpose of this study was to explore the associations between FNT kinematic variables obtained via Inertial Measurement Unit and multilevel upper extremity motor function in subacute stroke survivors. Furthermore, we aimed to compare the amount of variance in clinical scales that could be explained by FNT kinematic variables. Hypothetically, kinematic metrics reflecting the UE movement strategy, smoothness, and velocity could be considered to measure more aspects of motor impairment (FMA-UE) than activity assessments (ARAT and MBI).

## 2. Materials and Methods

### 2.1. Study Design

This cross-sectional study followed the Strengthening the Reporting of Observational Studies in Epidemiology (STROBE) checklist. The study was performed in accordance with the principles of the Declaration of Helsinki. The study protocol was approved by the Clinical Trials Ethics Committee of Huazhong University of Science and Technology on 24 October 2018. The study was registered in the Chinese Clinical Trial Registry (no. ChiCTR1900026656) on 17 October 2019.

### 2.2. Participants

Thirty-seven individuals with subacute stroke were recruited from the Department of Rehabilitation Medicine from December 2019 to January 2021 (Figure 1). The inclusion criteria were as follows: (a) clinical diagnosis of unilateral, first-ever subacute stroke verified by MRI or CT; (b) aged 18–80 years; (c) showing upper limb motor impairment (Fugl-Meyer Assessment of Upper Extremity <66); (d) able to complete the kinematic protocol; (e) no complicating medical history, such as visual, cardiac, or pulmonary disorders. Those who had other musculoskeletal or neurological conditions that affected arm function were excluded from the study [23]. All the participants were right handed [26] and have provided written informed consent prior to study entrance.

### 2.3. Clinical Assessments

Clinical assessments of the participants included the Fugl-Meyer Assessment of Upper Extremity (FMA-UE), Action Research Arm Test (ARAT), and modified Barthel Index (MBI). The FMA-UE is a validated and reliable assessment of poststroke upper limb motor impairment. FMA-UE is composed of 33 items that comprise four subscales (arm, wrist, hand, and coordination) regarding motor domains, and higher scores indicate less motor impairment of upper extremity [27]. The ARAT was used to evaluate UE functional capacity, including grasp, grip, pinch, and gross movement. ARAT consists of 19 four-point ordinal items, and higher scores indicate greater arm functional capacity [28]. The independence level in basic activities of living was assessed with the MBI, which consists of 10 items and higher scores indicate greater ADL independence [29].

### 2.4. Kinematic Assessment

Kinematic assessment was implemented with an Inertial Measurement Unit system (IMU, Noraxon USA Inc.). Each IMU sensor contains a coordinate system to assess accelerations and three-dimensional orientations at a 100 Hz sampling frequency. The IMU system had shown excellent reliability, accuracy, and precision in quantifying kinematic test [17]. Four sensors were placed on body segments, including head, upper arm, forearm, and hand, to detect UE kinematic information. Participants were required to sit in a height-adjustable chair with their hips and knees flexed to 90°. Upper extremity maintained in the neutral position, with elbow extension and palm downward initially. Standardized procedure for the finger-to-nose test was first presented by the same researcher, and then, it was imitated by the participants for three times before testing. The tests were recorded for five times, and a mean of the variable was used in statistical calculations [30].

Data were extracted through a semiautomated code in MATLAB software (The MathWorks, Natick, Massachusetts, USA) according to the anatomical coordinate system and joint rotation recommended by the International Society Biomechanical (ISB) [31]. Onsets and ends of FNT movements were defined with a velocity threshold of 50 mm/s [30]. In this cross-sectional study, six FNT kinematic variables were calculated: movement time (MT), mean velocity (VM), peak velocity (VP), percentage of time to peak velocity (TVP%), number of movement units (NMU), and normalized integrated jerk (NIJ) [30, 32]. MT was an objective quantitative variable defined as the time spent during the test to reflect movement performance. The maximum tangential velocity of index finger was calculated during each movement segment to get VP; VM was defined as the average tangential velocity. TVP% was the proportion of time taken from the onset of the movement to the peak velocity. The number of velocity peaks exceeding 10% of VP was characterized as NMU. NIJ was utilized to assess movement smoothness, which was calculated using jerk, M,T and length of the task according to the following formula:

(1) $$\begin{array}{c} \text{NIJ}=\;\sqrt{\frac{{\text{MT}}^{5}}{2\times {\text{length}}^{2}}\times \sum \text{jerk}{\left(t\right)}^{2}}, \end{array}$$

where jerk represented the third derivate of end point displacement, and length represented the shortest distance between initial and terminal positions of index finger.

### 2.5. Statistical Analysis

Statistical analysis was performed on IBM Statistical Package for Social Science (SPSS) version 22.0. Chi-squared test was used to examine categorical variables, and one-way ANOVA was used to examine quantitative variables. Shapiro–Wilk test or Q-Q plot was used to evaluate whether the quantitative data were normally distributed. Pearson's correlation coefficients (*r*) were conducted between kinematic and clinical assessments. The limit for multicollinearity among independent variables was set at 0.7 for correlation coefficients. After controlling the influencing factors (including age, gender, type of stroke, and paretic side), the kinematic metrics were included as independent variables into the multivariable linear regression to investigate the associations with clinical assessments. Probability for entry in backward regression was set at 0.05 and removal at 0.10. Adjusted *R*^2^ values with *P* value, unstandardized coefficient (*β*), and unique partial correlation coefficients were used to estimate the contribution of each metrics to the models. A two-sided *P* < 0.05 was set as statistical significance.

## 3. Results

### 3.1. Demographics and Clinical Characteristics

Demographics and clinical characteristics of the participants are presented in Table 1. Thirty-seven individuals (28 male, aged 49.78 ± 10.26 years) with subacute stroke were recruited in this study from December 2019 to January 2021 (Figure 1). They had moderate-to-severe UE motor impairment (mean FMA-UE scores, 36.22 ± 17.69) and capacity (mean ARAT scores, 23.97 ± 17.38). Of the 37 participants, 26 (70.3%) had ischemic stroke and 11 (29.7%) had hemorrhagic stroke; 22 (59.5%) had left-sided hemiplegia and 15 (40.5%) had right-sided hemiplegia (Table 1).

### 3.2. Correlations between Clinical and Kinematic Measures

Correlations between clinical and kinematic measures are shown in Table 2. Mean velocity strongly correlated with the FMA-UE (*r* = 0.85, *P* < 0.01) and ARAT (*r* = 0.80, *P* < 0.01) and moderately correlated with MBI positively (*r* = 0.58, *P* < 0.01). Besides, all the clinical assessments correlated significantly with VP positively (*r* = 0.55 to 0.81, *P* < 0.01) and NMU negatively (*r* = −0.45 to −0.65, *P* < 0.05). However, MT, TVP%, and NIJ were not significantly associated with the clinical assessments (Table 2). As shown in Table 2, multicollinearities were observed between MT and NIJ, as well as among VM, VP, and NMU. For that reason, only the VM and NIJ/MT during the FNT task were inputted into the multivariable linear regression models to estimate variation in clinical assessments.

The results of multivariable regression analysis of the kinematic metrics against the clinical assessments are presented in Table 3. Backward multiple regression revealed that kinematic variables could explain the largest amount of variance in the assessment of UE motor impairment as measured by FMA-UE. The only significant predictor was the VM, which explained 55% of the FMA-UE variance (*F* = 20.72, *P* < 0.01). Moreover, the VM alone showed a significant contribution to the models, accounting for 51% of the ARAT variance (*F* = 39.10, *P* < 0.01) and 32% of the MBI variance (*F* = 8.93, *P* < 0.01) (Table 3). Moreover, demographics, including age, gender, type of stroke, and paretic side, showed no significant influence in any regression model.

## 4. Discussion

The cross-sectional study investigated the associations between FNT kinematic variables obtained via Inertial Measurement Unit and upper extremity motor function in subacute stroke survivors according to the ICF framework. The results indicated that the mean velocity (*r* = 0.58 to 0.85), peak velocity (*r* = 0.55 to 0.81), and number of movement units (*r* = −0.45 to −0.65) were associated with all of the clinical assessments. Mean velocity was entered into the multivariable linear regression models and could estimate 55%, 51%, and 32% of variance in FMA-UE, ARAT, and MBI during the FNT task. Additionally, age, gender, type of stroke, and paretic side had no significant effects on these associations.

The previous kinematic literature mainly focused on predicting upper limb motor impairment. Our results extended the value of kinematic scenarios beyond the impairment level according to the ICF framework and suggested that FNT kinematics was more strongly associated with FMA-UE and ARAT than MBI. Lee et al. proposed an automated FMA system and showed high scoring accuracy in 79% of FMA test in nine stroke patients [33]. Their algorithms were shown appropriate for clinical use but lacked clinical interpretability in kinematic results because estimating clinical scale was not the only goal of portable sensors [14, 16, 34]. In addition, little was known about the associations between clinical activity–related scales and IMU sensors [35]. Our models established predictable correlations between FNT mean velocity via Inertial Measurement Unit and upper extremity motor function after stroke [36].

Due to multicollinearity among VM, VP, and NMU, only VM was entered into the multivariable models. Speed variables reflect how efficiently a person controls interaction torques of the agonist/antagonist muscles [32]. Analogous to our results, two studies using robotic device showed significant correlations between movement speed and FMA-UE in individuals with subacute [37] and chronic [38] stroke, respectively. Furthermore, movement smoothness is an important indicator of upper limb motor recovery after stroke [30]. Smoothness parameters evaluate the temporal organization or UE multijoint coordination [39]. In a study early after stroke, smoothness measured by NMU was able to predict upper limb motor recovery over time [40]. According to our results, NIJ was not significantly associated with the clinical assessments. However, smoothness should be interpreted with cautions because a single smoothness parameter may not completely reflect motor recovery of upper extremity [41].

Interestingly, the FNT kinematic metrics measured comparable aspects of motor impairment by FMA-UE (*R*^2^ = 0.55) and functional capacity by ARAT (*R*^2^ = 0.51). This was analogous with a prior work by Adans-Dester et al., which used eight motor tasks of Wolf Motor Function Test (WMFT) and found satisfactory results to estimate upper limb impairment and activity scales [42]. Although this was in line with our second hypothesis, the difference was small and needed to be further studied [19]. One possible explanation might be that participants had moderate-to-severe upper extremity motor impairment, leading to poor scores on manual dexterity of ARAT items. Future studies should therefore include much kinematic variables and comprehensive tasks at different UE segments to explore the correlations between the assessments. The low variance explained by IMU kinematic variables in MBI could be that the FNT task did not measure distal dexterity of the upper extremity. As a result, variables in the models may not fully capture kinematic information in individuals with stroke [43]. Moreover, MBI is a questionnaire for ADL in a real environment and not an observational measure of UE motor function in an experimental setting. Thus, participants could use compensatory behaviors or actually the less affected UE to improve MBI scores, which may be difficult to explain with the current kinematic task.

Several limitations of this study should be acknowledged. First, the sample size restricted the number of kinematic variables entered into the multivariable linear regression models. Therefore, future studies could implement other statistical models, such as machine-learning approaches, to investigate the associations between FNT kinematic variables and upper extremity motor function in individuals with stroke [42, 44]. Second, this was a cross-sectional study and unable to investigate the longitudinal associations between kinematics and clinical measurements. Finally, the models did not include other kinematic tests and variables concerning trunk and interjoint movements, which may lead to task-related bias and loss of information [45, 46].

## 5. Conclusions

This study indicates that kinematic variables measured via Inertial Measurement Unit during the finger-to-nose task are associated with upper extremity motor function in individuals with subacute stroke according to the ICF framework. Furthermore, the objective kinematic evaluation may be suitable for predicting clinical measures of motor impairment and capacity to understand upper extremity motor recovery and clinical decision making after stroke.

## Figures and Tables

**Figure 1:** Flowchart of the study.

**Table 1:** Demographics and clinical characteristics (*n* = 37).

Characteristics (*n* = 37)	
Age (years)	49.78 ± 10.26
Gender (M/F)	28/9
Days between onset and enrollment	106.30 ± 65.46
Type of stroke (ischemic/hemorrhagic)	26/11
Paretic side (left/right)	22/15
FMA-UE (range 0–66)	36.22 ± 17.69
ARAT (range 0–57)	23.97 ± 17.38
MBI (range 0–100)	72.30 ± 22.20
Body mass index (kg/m^2^)	24.43 ± 2.60
MT (s)	1.09 ± 0.31
VP (m/s)	1.61 ± 0.92
VM (m/s)	0.78 ± 0.44
TVP% (%)	42.23 ± 11.30
NMU	2.56 ± 1.25
NIJ	2.86 ± 1.98

FMA-UE, Fugl-Meyer assessment for upper extremity; ARAT, action research arm test; MBI, Modified Barthel index; MT: movement time; VP: peak velocity; VM: mean velocity; TVP%: percentage of time to peak velocity; NMU: Number of movement units; NIJ: Normalized integrated jerk.

**Table 2:** Correlations between clinical assessments and kinematic metrics (*n* = 37).

	FMA	ARAT	MBI	MT	VP	VM	TVP%	NMU
*Clinical assessment*								
FMA								
ARAT	0.94^*∗∗*^							
MBI	0.62^*∗∗*^	0.64^*∗∗*^						

*Kinematic metrics*								
MT	0.11	0.07	0.15					
VP	0.81^*∗∗*^	0.76^*∗∗*^	0.55^*∗∗*^	−0.03				
VM	0.85^*∗∗*^	0.80^*∗∗*^	0.58^*∗∗*^	−0.11	0.96^*∗∗*^			
TVP%	−0.11	−0.17	−0.14	−0.49^*∗*^	−0.17	−0.11		
NMU	−0.65^*∗∗*^	−0.59^*∗∗*^	−0.45^*∗*^	0.10	−0.70^*∗∗*^	−0.74^*∗∗*^	0.22	
NIJ	−0.24	−0.27	−0.10	0.71^*∗∗*^	−0.27	−0.40^*∗∗*^	−0.20	0.47^*∗*^

FMA-UE, Fugl-Meyer Assessment for Upper xtremity; ARAT, Action Research Arm Test; MBI, Modified Barthel Index; MT: movement time; VP: peak velocity; VM: mean velocity; TVP%: percentage of time to peak velocity; NMU: Number of movement units; NIJ: Normalized integrated jerk. ^*∗*^: *P* < 0.05. ^*∗∗*^: *P* < 0.01.

**Table 3:** Multivariable regression analysis of the kinematic metrics against the clinical assessments (*n* = 37).

Independent variables	Unstandardized coefficient *β*	Standard error	Partial unique correlations	*P* value of the variable	Adjusted *R*^2^ (model *P* value)
*FMA-UE as dependent variable*					0.55 (<0.01^*∗*^)
Constant	11.91	2.59	—	<0.01^*∗*^	
VM	17.81	2.90	0.74	<0.01^*∗*^	
NIJ	1.05	0.68	0.25	0.13	

*ARAT as dependent variable*					0.51 (<0.01^*∗*^)
Constant	1.50	4.11	—	0.72	
VM	28.84	4.61	0.73	<0.01^*∗*^	

*MBI as dependent variable*					0.32 (0.01^*∗*^)
Constant	32.57	12.23	—	0.19	
VM	28.93	7.09	0.57	<0.01^*∗*^	
MT	15.70	10.05	0.26	0.13	

FMA-UE, Fugl-Meyer Assessment for Upper Extremity; ARAT, action research arm test; MBI, Modified Barthel Index; MT: movement time; VM: mean velocity; NIJ: normalized integrated jerk. ^*∗*^: *P* < 0.05.

## Data Availability

The data files are available from the corresponding author upon reasonable request.

## References

[1] Langhorne P., Coupar F., Pollock A. (2009). Motor recovery after stroke: a systematic review. *The Lancet Neurology*.

[2] Kwakkel G., Kollen B. J., van der Grond J., Prevo A. J. H. (2003). Probability of regaining dexterity in the flaccid upper limb. *Stroke*.

[3] Lloyd-Jones D., Adams R. J., Brown T. M. (2010). Heart disease and stroke statistics--2010 update: a report from the American Heart Association. *Circulation*.

[4] Stinear C. (2010). Prediction of recovery of motor function after stroke. *The Lancet Neurology*.

[5] Villepinte C., Verma A., Dimeglio C., De Boissezon X., Gasq D. (2020). Responsiveness of kinematic and clinical measures of upper-limb motor function after stroke: a systematic review and meta-analysis. *Annals of Physical and Rehabilitation Medicine*.

[6] Santisteban L., Térémetz M., Bleton J.-P., Baron J.-C., Maier M. A., Lindberg P. G. (2016). Upper limb outcome measures used in stroke rehabilitation studies: a systematic literature review. *PLoS One*.

[7] Lang C. E., Bland M. D., Bailey R. R., Schaefer S. Y., Birkenmeier R. L. (2013). Assessment of upper extremity impairment, function, and activity after stroke: foundations for clinical decision making. *Journal of Hand Therapy*.

[8] Schwarz A., Bhagubai M. M. C., Wolterink G., Held J. P. O., Luft A. R., Veltink P. H. (2020). Assessment of upper limb movement impairments after stroke using wearable inertial sensing. *Sensors*.

[9] Grimm F., Kraugmann J., Naros G., Gharabaghi A. (2021). Clinical validation of kinematic assessments of post-stroke upper limb movements with a multi-joint arm exoskeleton. *Journal of NeuroEngineering and Rehabilitation*.

[10] Chen Z. J., He C., Guo F., Xiong C. H., Huang X. L. (2021). Exoskeleton-assisted anthropomorphic movement training (eamt) for post-stroke upper limb rehabilitation: a pilot randomized controlled trial. *Archives of Physical Medicine and Rehabilitation*.

[11] Balasubramanian S., Colombo R., Sterpi I., Sanguineti V., Burdet E. (2012). Robotic assessment of upper limb motor function after stroke. *American Journal of Physical Medicine and Rehabilitation*.

[12] Johansson G. M., Grip H., Levin M. F., Häger C. K. (2017). The added value of kinematic evaluation of the timed finger-to-nose test in persons post-stroke. *Journal of NeuroEngineering and Rehabilitation*.

[13] Hughes C. M. L., Baye M., Gordon-Murer C. (2019). Quantitative assessment of upper limb motor function in Ethiopian acquired brain injured patients using a low-cost wearable sensor. *Frontiers in Neurology*.

[14] Maceira-Elvira P., Popa T., Schmid A.-C., Hummel F. C. (2019). Wearable technology in stroke rehabilitation: towards improved diagnosis and treatment of upper-limb motor impairment. *Journal of NeuroEngineering and Rehabilitation*.

[15] Who I. C. F. (2001). *International Classification of Functioning, Disability and Health*.

[16] Oubre B., Daneault J.-F., Jung H.-T. (2020). Estimating upper-limb impairment level in stroke survivors using wearable inertial sensors and a minimally-burdensome motor task. *IEEE Transactions on Neural Systems and Rehabilitation Engineering*.

[17] Öhberg F., Bäcklund T., Sundström N., Grip H. (2019). Portable sensors add reliable kinematic measures to the assessment of upper extremity function. *Sensors*.

[18] Lee S., Lee Y.-S., Kim J. (2018). Automated evaluation of upper-limb motor function impairment using fugl-meyer assessment. *IEEE Transactions on Neural Systems and Rehabilitation Engineering*.

[19] Del Din S., Patel S., Cobelli C., Bonato P. (2011). Estimating Fugl-Meyer clinical scores in stroke survivors using wearable sensors. *Annu Int Conf IEEE Eng Med Biol Soc*.

[20] Schwarz A., Kanzler C. M., Lambercy O., Luft A. R., Veerbeek J. M. (2019). Systematic review on kinematic assessments of upper limb movements after stroke. *Stroke*.

[21] Tran H., Nguyen K. D., Pathirana P. N., Horne M. K., Power L., Szmulewicz D. J. (2020). A comprehensive scheme for the objective upper body assessments of subjects with cerebellar ataxia. *Journal of NeuroEngineering and Rehabilitation*.

[22] Otten P., Kim J., Son S. (2015). A framework to automate assessment of upper-limb motor function impairment: a feasibility study. *Sensors*.

[23] Rodrigues M. R. M., Slimovitch M., Chilingaryan G., Levin M. F. (2017). Does the Finger-to-Nose Test measure upper limb coordination in chronic stroke?. *Journal of NeuroEngineering and Rehabilitation*.

[24] Chen W., Xiong C., Huang X., Sun R., Xiong Y. (2010). Kinematic analysis and dexterity evaluation of upper extremity in activities of daily living. *Gait & Posture*.

[25] Liu K., Xiong C.-H., He L., Chen W.-B., Huang X.-L. (2018). Postural synergy based design of exoskeleton robot replicating human arm reaching movements. *Robotics and Autonomous Systems*.

[26] Verdino M., Dingman S. (1998). Two measures of laterality in handedness: the Edinburgh Handedness Inventory and the Purdue Pegboard test of manual dexterity. *Perceptual & Motor Skills*.

[27] See J., Dodakian L., Chou C. (2013). A standardized approach to the Fugl-Meyer assessment and its implications for clinical trials. *Neurorehabilitation and Neural Repair*.

[28] Van der Lee J. H., De Groot V., Beckerman H., Wagenaar R. C., Lankhorst G. J., Bouter L. M. (2001). The intra- and interrater reliability of the action research arm test: a practical test of upper extremity function in patients with stroke. *Archives of Physical Medicine and Rehabilitation*.

[29] Hsieh Y.-W., Wang C.-H., Wu S.-C., Chen P.-C., Sheu C.-F., Hsieh C.-L. (2007). Establishing the minimal clinically important difference of the Barthel Index in stroke patients. *Neurorehabilitation and Neural Repair*.

[30] Schiefelbein M. L., Salazar A. P., Marchese R. R. (2019). Upper-limb movement smoothness after stroke and its relationship with measures of body function/structure and activity - a cross-sectional study. *Journal of the Neurological Sciences*.

[31] Wu G., van der Helm F. C. T., Veeger H. E. J. (2005). ISB recommendation on definitions of joint coordinate systems of various joints for the reporting of human joint motion-Part II: shoulder, elbow, wrist and hand. *Journal of Biomechanics*.

[32] Nordin N., Xie S., Wünsche B. (2014). Assessment of movement quality in robot- assisted upper limb rehabilitation after stroke: a review. *Journal of NeuroEngineering and Rehabilitation*.

[33] Park E., Lee K., Han T., Nam H. S. (2020). Automatic grading of stroke symptoms for rapid assessment using optimized machine learning and 4-limb kinematics: clinical validation study. *Journal of Medical Internet Research*.

[34] Nelson Z., Wade E. (2018). Relative efficacy of sensor modalities for estimating post-stroke motor impairment. *Annual International Conference of the IEEE Engineering in Medicine and Biology Society. IEEE Engineering in Medicine and Biology Society. Annual International Conference*.

[35] Li J., Pan B., Jin T. (2016). A single task assessment system of upper-limb motor function after stroke. *Technology and Health Care*.

[36] Hussain N., Sunnerhagen K. S., Alt Murphy M. (2021). Recovery of arm function during acute to chronic stage of stroke quantified by kinematics. *Journal of Rehabilitation Medicine*.

[37] Duret C., Courtial O., Grosmaire A. G. (2016). Kinematic measures for upper limb motor assessment during robot-mediated training in patients with severe sub-acute stroke. *Restorative Neurology and Neuroscience*.

[38] Zollo L., Gallotta E., Guglielmelli E., Sterzi S. (2011). Robotic technologies and rehabilitation: new tools for upper-limb therapy and assessment in chronic stroke. *European Journal of Physical and Rehabilitation Medicine*.

[39] Balasubramanian S., Melendez-Calderon A., Roby-Brami A., Burdet E. (2015). On the analysis of movement smoothness. *Journal of NeuroEngineering and Rehabilitation*.

[40] van Dokkum L., Hauret I., Mottet D., Froger J., Métrot J., Laffont I. (2014). The contribution of kinematics in the assessment of upper limb motor recovery early after stroke. *Neurorehabilitation and Neural Repair*.

[41] Rohrer B., Fasoli S., Krebs H. I. (2002). Movement smoothness changes during stroke recovery. *Journal of Neuroscience*.

[42] Adans-Dester C., Hankov N., O’Brien A. (2020). Enabling precision rehabilitation interventions using wearable sensors and machine learning to track motor recovery. *Npj Digital Medicine*.

[43] Bosecker C., Dipietro L., Volpe B., Igo Krebs H. (2010). Kinematic robot-based evaluation scales and clinical counterparts to measure upper limb motor performance in patients with chronic stroke. *Neurorehabilitation and Neural Repair*.

[44] Chen Z.-J., He C., Xia N. (2021). Association between finger-to-nose kinematics and upper extremity motor function in subacute stroke: a principal component analysis. *Frontiers in Bioengineering and Biotechnology*.

[45] Schwarz A., Veerbeek J. M., Held J. P. O., Buurke J. H., Luft A. R. (2020). Measures of interjoint coordination post-stroke across different upper limb movement tasks. *Frontiers in bioengineering and biotechnology*.

[46] Kim G. J., Parnandi A., Eva S., Schambra H. (2021). The use of wearable sensors to assess and treat the upper extremity after stroke: a scoping review. *Disability & Rehabilitation*.

